The article "A Survey Study on the Status of Somatic Symptoms in Young and Middle-Aged Patients with Mental Illness during Long-Term Hospitalization" was published in 2022. Journal: Contrast Media Mol Imaging.

# A Survey Study on the Status of Somatic Symptoms in Young and Middle-Aged Patients with Mental Illness during Long-Term Hospitalization

**DOI:** 10.1155/2022/1110941

**Published:** 2022-07-20

**Authors:** Wenxin Zheng, Zhiwei Guo

**Affiliations:** ^1^Chongqing Medical University Mental Medical Discipline, Chongqing 400016, China; ^2^Department of Cardiovascular Medicine, Hangzhou Ninth People's Hospital, Hangzhou 310020, China

## Abstract

Psychiatric disorders include severe psychiatric disorders and those in general with some psychiatric disorders having a clear etiology or in which a significant psychiatric predisposing factor is present. Whereas, psychiatric disorders precisely refer to those characterized by mild depression and mild anxiety and appear to affect a large number of people in any community. It has been reported that the disease is highly prevalent and has a huge impact on the individual, family, and community levels, resulting in a heavy burden on the healthcare system of a country. To explore the status of somatic symptoms in young and middle-aged psychiatric patients during long-term hospitalization, a total of 114 young and middle-aged psychiatric patients with prolonged hospitalization (more than 5 years) were included. Data information of the hospitalized patients was recorded, including preadmission somatic symptoms, electrocardiogram (ECG), echocardiogram, abdominal ultrasound, and blood tests. In addition, a homemade questionnaire was administered, and general information about the patients was also collected, including gender, age, current medication use, and duration of medication use. Correlations between cardiometabolic disease, osteoporosis, and long-term oral antipsychotic medication were analyzed in these young and middle-aged patients. The prevalence of comorbid somatic symptoms was 77.2%, and concomitant disorders included mainly cardiometabolic disorders, osteoporosis, pulmonary infections, cerebrovascular disorders, digestive disorders, fractures, and skin conditions. The incidence of somatic symptoms caused by long-term use of antipsychotic drugs was about 88.6%, and the incidence of concomitant somatic symptoms was higher in young and middle-aged psychiatric patients who were hospitalized for a long time. The current study observed a high prevalence of somatic symptoms in young and middle-aged patients with long-term inpatient psychiatric illness. Endocrine and metabolic disorders, particularly dyslipidemia, may trigger a range of deleterious effects. In addition to this, there is a high incidence of osteoporosis. Special attention should be paid to the side effects of antipsychotic drugs, and appropriate measures are needed to make early diagnosis and provide early treatment to reduce the occurrence of cardiometabolic diseases and osteoporosis.

## 1. Introduction

Mental illness, those disorders that are characterized by a combination of mild depression, mild anxiety, and medically unexplained physical symptoms, seem to affect a significant number of people in any community. Such disorders are reported to be highly prevalent and have a huge impact at the individual, family, and community levels [1, 2], causing a significant burden on a country's healthcare system [3, 4].

Somatic symptoms related to emotional difficulties are frequent presentations in general practice and have been estimated to account for more than half of all outpatient encounters [5, 6], are medically unexplained, and are purely due to psychological distress or health-seeking behavior that may be present in at least 10–15% of all primary care patients [7, 8]. Somatic symptoms may be high in primary care patients for various reasons, such as panic disorder patients who present with somatic complaints, depression, or other disorders [9, 10].

In China, the incidence of affective disturbance is rising and is consequently becoming an important health challenge. A study showed that the rate of anxiety was 71.2%, the rate of depression was 64.7%, and the rate of somatic complaints was 64.9% [11]. However, the prevalence of somatic symptoms in China, especially in patients who were present at clinics or general hospitals, has not been well studied, and little attention has been given to the correlation of somatic symptoms with young and middle-aged long-term hospitalized patients with mental illnesses [12].

Therefore, we conducted a two-year survey over the somatic symptoms of patients with chronic mental illness who had stayed in the hospital for five years or more to investigate the status of the somatic symptoms in young and middle-aged psychiatric patients in long-term hospitalization.

## 2. Methods

### 2.1. Study Population

The patients with mental illness who had stayed in the hospital for over five years were included.

Inclusion criteria were as follows: (1) patients who were conformed to the diagnostic criteria for schizophrenia and mental retardation (according to the Chinese Classification and Diagnosis of Mental Disorders, Fourth Edition, CCMD-10). Diagnostic criteria for schizophrenia—symptoms less than 2 of the following criteria: recurrent verbal hallucinations; marked laxity, disrupted thinking, incoherent speech, poor thinking, or lack of thought content; thinking is inserted, withdrawn, disseminated, disrupted, or mandatory; passive, controlled, or given insight into the experience; primary delusions (including delusional perceptions and delusional mood) or other paranoid delusions; thinking logically fell short, pathologically symbolic thinking, or a new work of words; apathy or marked apathy; tension syndrome, bizarre behavior, or woolly behavior; and marked reduction or lack of volition; (2) patients who had stayed in the hospital for five years or more; and (3) patients who had no somatic symptoms before admission; (4) patients and their relatives who were willing to cooperate with the treatment regimen and signing the informed consent form. Exclusion criteria were as follows: (1) patients who had severe somatic and organic diseases, including a personal and family history of hypertension, cardiovascular diseases, adrenal and thyroid diseases, and personal history of syphilis; (2) patients with drug allergy; (3) patients with alcohol and drug dependence; (4) pregnant and lactating women; (5) patients without antipsychotics treatment; (6) patients with abnormalities found upon blood tests and ECG before the admission; and (7) patients with an unclear diagnosis. The project received institutional research ethics board approval before the beginning of the study from the Authority Research Ethics Board, No. 2022-000-J025.

### 2.2. Clinical Data Collection

Inpatient medical records were reviewed. Somatic symptoms, ECG, echocardiography, abdominal ultrasound, and blood tests before admission were reviewed. The patients were surveyed using a self-made questionnaire. The patients' general information was collected, including gender, age, current medications, and duration of the medication. Current medications mainly consisted of the following: risperidone, olanzapine, quetiapine fumarate, ziprasidone, aripiprazole, clozapine, perphenazine, sulpiride, SSRI and SNRI antidepressants, lithium carbonate, benzodiazepines, and antiepileptic drugs.

### 2.3. Examination

The standard 12-lead ECG was performed with a 25 mm/s paper speed and a standard voltage set to 0 mm = l mv. ECG was administered at least once or twice upon admission and every 4 w after the treatment began. Abnormal ECG changes, such as QTc interval and ST-T changes, were monitored. The bone density test was performed once every 4–8 w after admission. Abdominal ultrasound, echocardiography, and thyroid ultrasound were performed once every 4–12 w after admission.

Blood tests, including the routine blood test, biochemistry test, and immunological test, were performed once or twice every 4–8 w after admission. The blood lipid profile, blood glucose, liver functions, and blood levels of homocysteine, prolactin, and thyroid hormones were evaluated. Blood pressures were measured and recorded at different time points and in erect and recumbent positions.

### 2.4. Statistical Analysis

All data analyses were conducted using IBM SPSS Statistics for Windows, version 27.0 (IBM Corporation, Armonk, NY, USA). The data are presented as the mean ± standard deviation. Plots were generated using Prism 7.0 software (GraphPad Software, Inc., San Diego, CA, USA).

## 3. Results

### 3.1. Basic Characteristics

A total of 247 patients with mental illness who had stayed in the hospital for over five years were surveyed. Among them, 145 young and middle-aged patients had no somatic symptoms before hospitalization. Other 102 elderly patients were combined with somatic symptoms or somatic symptom-induced mental disorders. Totally, 114 patients who met the inclusion and exclusion criteria were included in the final analysis. There were 83 males and 31 females meeting the diagnostic criteria. There were 6 patients in the young adult group and 108 patients in the middle-aged group. These patients were aged 49.07 ± 7.30 years old, with a course of disease ≥5 years. They were taking antipsychotics orally (1–5 types of antipsychotics).

As for the type of mental illness, there were 96 patients with schizophrenia and 15 patients with mental retardation. Five patients were taking conventional antipsychotics, 6 patients were taking conventional antipsychotics plus atypical antipsychotics, 59 patients were taking one type of atypical antipsychotics, and 44 patients were taking two or more types of atypical antipsychotics.

### 3.2. Common Concomitant Somatic Symptoms

There were 88 patients combined with somatic symptoms, accounting for 77.2%.  Figure 1 shows the percentage of patients with cardiometabolic diseases.  Figure 2 shows the percentage of patients with digestive diseases. As shown in Figure 1, dyslipidemia was present in 85% of 88 cases in patients with cardiometabolic diseases, hyperhomocysteinemia in 40%, 15% with high blood glucose, hypertension in 8%, and arrhythmias in 3%. As shown in Figure 2, gallbladder diseases accounted for 9% of the patients with digestive diseases, gastrointestinal dysfunction in 7%, fatty liver in 14%, and liver damage in 7%.

Acute concomitant somatic symptoms included respiratory tract infection and intestinal infection in 21 patients, arrhythmia in 3 patients, trauma caused by poor management in 5 patients, intestinal obstruction in 3 patients, gastrointestinal bleeding in 2 patients, a hyperosmolar hyperglycemic state in 1 patient, and chicken pox in 1 patient. While for chronic somatic symptoms, it was found that dyslipidemia was present in 93 patients, hyperhomocysteinemia in 46 patients, osteoporosis in 34 patients, hypertension in 18 patients, hyperprolactinemia in 18 patients, hypothyroidism in 18 patients, kidney stones in 16 patients, fatty liver in 16 patients, gallbladder disorders (including gallstones and gallbladder polyps) in 11 patients, type 2 diabetes in 10 patients, abnormal glucose tolerance in 8 patients, gastrointestinal dysfunction in 8 patients, liver damage in 7 patients, anemia in 4 patients, arrhythmias in 3 patients (ventricular premature beats in 1 patient, atrial premature beats in 1 patient, and atrial fibrillation in 1 patient), skin conditions in 3 patients, hyperuricemia in 2 patients, cirrhosis with or without complications in 1 patient, electrolyte disturbances in 2 patients, and abnormal white blood cell count in 5 patients.  Table 1 provides the baseline data of somatic symptoms in the included patients.

Cardiometabolic diseases include dyslipidemia, hyperglycemia, hypertension, arrhythmias, and hyperhomocysteinemia. Digestive diseases include gastrointestinal dysfunction, intestinal obstruction, gallbladder diseases, and fatty liver. Urinary system diseases include kidney stones and hydronephrosis.

## 4. Discussion

The current study has observed a high prevalence of somatic symptoms in young and middle-aged long-term hospitalized patients with mental illnesses. Endocrine and metabolic disorders, especially dyslipidemia, may trigger a cascade of harmful effects. Apart from that, the incidence of osteoporosis is also high.

The cascade of adverse metabolic effects starts with increased appetite and weight gain and progressively evolves to obesity, insulin resistance, and elevated levels of cholesterol and triglycerides. The patients suffering from dyslipidemia and hyperinsulinemia finally develop into the damage of islet *β*-cells and prediabetes [13]. Then, diabetes further increases the risk of cardiovascular events and premature death [14]. A high triglyceride level combined with insulin resistance caused by antipsychotics may also increase cardiometabolic risk [15].

It is necessary to monitor patients taking antipsychotics and manage the cardiometabolic risk. If there is a significant increase in BMI or fasting triglycerides, a change to the kind of antipsychotics that will not cause the above problems may be considered. The atypical antipsychotics were reported to be related to weight gain and cardiometabolic diseases [16]. Therefore, antipsychotics should be selected appropriately based on various monitoring indicators to reduce cardiometabolic risk and premature death. If the patients are already combined with diabetes, hyperlipidemia, prediabetes, or diabetes, blood pressure monitoring, rapid blood glucose testing, and waist circumference measurement are important during the antipsychotic treatment.

All subjects in this study were young and middle-aged patients who were of 60 years or above. The occurrence of osteoporosis is related to many factors, and hormones are important factors. Among various hormones, a high prolactin level plays an indispensable role. An elevation of the serum prolactin level combined with hypogonadism can inhibit the secretion of gonadotropin-releasing hormone (GnRH). A low GnRH level will cause a reduction in luteinizing hormone (LH) and follicle-stimulating hormone (FSH) secreted by the pituitary gland. As a result, estradiol, progesterone, and testosterone are secreted in lesser amounts. The reduction in these hormones will finally increase osteoclast activity. Moreover, the osteoclast activity outweighs the osteoblast activity, leading to the abnormal bone metabolism similar to type I osteoporosis [17, 18]. It has been shown that on the molecular level, prolactin receptors can be found in human osteoblasts. Prolactin can directly reduce osteoblast proliferation, causing the number of osteoblasts to decrease. The osteoblast activity decreases correspondingly, while the osteoclast activity is enhanced, which reduces the bone density [19, 20].

Psychiatric disorders, due to epilepsy, account for a high proportion of psychiatric disorders, and patients have a long disease duration and high recurrence rate, and studies have shown that patient prognosis is affected by maintenance treatment and the recovery of social function. Now that most patients are treated in the hospital and their condition is stable enough to be discharged home, continued treatment after discharge, along with care, is also crucial. Therefore, in addition to requiring patients to be able to take their medication regularly, there is a need to provide nursing services that allow patients to have a reduced chance of recurrence and facilitate recovery [17]. The disease belongs to the group of once ill, life-long diseases, and will recur; our mental health resources are lacking, and the rational use of drugs in the clinic can allow the patient's condition to be significantly improved; in addition, combination therapy, when it is necessary to provide psychological care, dietary care, rehabilitation care, and other nursing measures, which can improve the therapeutic effect, especially psychological care, is very important in the whole process of care. The medication adherence of patients has significantly improved and is a very important factor in the clinical treatment of patients.

The combined use of antiepileptics as mood stabilizers is a common treatment for mental illnesses. The long-term use of antiepileptics has various effects on bone density and bone metabolism. Among the studies on the effects of antiepileptics on the bone density and bone metabolism, the liver enzyme inducer has been considered an important factor [21–23]. Some antiepileptics act as liver enzyme inducers, which induce hepatic cytochrome P450, accelerating vitamin D metabolism and decreasing the vitamin D level. Hence, bone metabolism disorders occur, and bone density decreases. VPA is a hepatic enzyme inhibitor, though it is believed to reduce bone density in many studies [24]. Therefore, disorders of bone formation occur, which is accompanied by bone mass reduction [25]. SSRIs, inhibitors of 5-HT reuptake, and 5-HT2 receptor antagonists may cause hyponatremia. Na + will be released from the bones in case of persistently low sodium levels [26, 27]. Holm et al. [28] reported that under a persistent low sodium level, osteoclast activity was increased, with more Na^+^ released from the bones. The release of Na^+^ from the bone matrix is achieved by osteoclasts promoting bone resorption, which further promotes Na^+^ balance in blood. This action is highly similar to the release of Ca^+^ from the bones in hypocalcemia [29]. Therefore, osteoclast-mediated bone resorption can cause a progressive bone density reduction, reducing the risks of osteoporosis and bone fractures.

## 5. Conclusion

The prevalence of somatic symptoms in young and middle-aged psychiatric patients with long-term hospitalization is very high. Psychiatrists should pay timely attention to the changes in patients' conditions through physical examination and conduct the regular auxiliary examination. Early diagnosis and treatment should be performed to prevent the occurrence of cardiometabolic diseases and osteoporosis.

## Figures and Tables

**Figure 1:** Percentage of patients with cardiometabolic diseases.

**Figure 2:** Percentage of patients with digestive diseases.

**Table 1:** Baseline data of somatic symptoms in the included patients.

Somatic symptoms	Cases	Age	Females	Males	BMI
Cardiometabolic diseases	100	49.3 ± 6.93	27	73	23.73 ± 3.45
Digestive diseases	42	49.2 ± 7.61	4	38	24.11 ± 3.69
Osteoporosis	37	49.4 ± 6.34	4	33	22.98 ± 3.63
Urinary system diseases	21	50.2 ± 8.07	2	19	24.52 ± 3.89
Thyroid diseases	17	50.5 ± 6.33	0	17	23.92 ± 4.08
Hyperprolactinemia	23	46.5 ± 8.37	8	15	23.17 ± 3.25

## Data Availability

The data used to support the findings of this study are available from the corresponding author upon request.
